# Automatic Detection of Cracks in Cracked Tooth Based on Binary Classification Convolutional Neural Networks

**DOI:** 10.1155/2022/9333406

**Published:** 2022-09-19

**Authors:** Juncheng Guo, Yuyan Wu, Lizhi Chen, Guanghua Ge, Yadong Tang, Wenlong Wang

**Affiliations:** ^1^School of Mechanical and Electrical Engineering, Guangzhou University, Guangzhou 510006, China; ^2^Department of Dentistry, Hospital of Guangdong University of Technology, Guangdong University of Technology, Guangzhou 510006, China; ^3^School of Biomedical and Pharmaceutical Sciences, Guangdong University of Technology, Guangzhou 510006, China

## Abstract

Cracked tooth syndrome is a commonly encountered disease in dentistry, which is often accompanied by dramatic painful responses from occlusion and temperature stimulation. Current clinical diagnostic trials include traditional methods (such as occlusion test, probing, cold stimulation, etc.) and X-rays based medical imaging (periapical radiography (PR), cone-beam computed tomography (CBCT), etc.). However, these methods are strongly dependent on the experience of the clinicians, and some inconspicuous cracks are also extremely easy to be overlooked by visual observation, which will definitely affect the subsequent treatments. Inspired by the achievements of applying deep convolutional neural networks (CNNs) in crack detection in engineering, this article proposes an image-based crack detection method using a deep CNN classifier in combination with a sliding window algorithm. A CNN model is designed by modifying the size of the input layer and adding a fully connected layer with 2 units based on the ResNet50, and then, the proposed CNN is trained and validated with a self-prepared cracked tooth dataset including 20,000 images. By comparing validation accuracy under seven different learning rates, 10^−5^ is chosen as the best learning rate for the following testing process. The trained CNN is tested on 100 images with 1920 × 1080-pixel resolutions, which achieves an average accuracy of 90.39%. The results show that the proposed method can effectively detect cracks in images under various conditions (stained, overexplosion, images affected by other diseases). The proposed method in this article provides doctors with a more intelligent diagnostic solution, and it is not only suitable for optical photographs but also for automated diagnosis of other medical imaging images.

## 1. Introduction

Cracked tooth syndrome, was defined as an incomplete fracture of the anterior molar, and it was considered as one of the major causes of tooth loss in adults [1, 2]. Later on, the American Association of Endodontists (AAE) divided cracked teeth into five types: craze lines, fractured cusp, cracked tooth, split tooth, and vertical root fracture (VRF) [3]. The diagnosis of a cracked tooth is a very challenging task, especially in the early stage, because it is extremely easy to be misdiagnosed due to indiscoverable microcracks and inconspicuous clinical symptoms [4]. The accurate diagnosis of cracked teeth is of great importance because it may influence the treatment strategy. On the other hand, it is difficult to make a definitive diagnosis based on signs and symptoms alone, because these signs and symptoms are nonspecific and similar to the clinical manifestations of endodontic and periodontal diseases. If the cracked tooth cannot be treated properly, the cracks would continue to expand and eventually cause pulpitis and even fracture of the entire tooth [5].

Usually, the diagnosis of a cracked tooth is mainly based on clinical symptoms [6]. For the suspected teeth, the clinician could determine them by several traditional clinical tests, such as the occlusion test method [7], probing method [8], cold stimulation method [9], light transillumination method [10], and so on. Currently, X-rays-based methods, especially CBCT, are widely applied in the clinical diagnosis of a cracked tooth, and many in vitro and in vivo studies have also validated the effect of CBCT in the diagnosis of VRF [11–14]. However, these available diagnosis methods may have some limitations. Methods like traditional clinical tests are not accurate enough, and they require a high level of clinician experience. Although transillumination and superficial dyes can make microfractures visible to the naked eye, the clinician's diagnostic decisions may be interfered due to visual fatigue. CBCT seems to be the crucial diagnostical solution. However, the doctors may misjudge the fracture and progression of the cracked tooth due to the impact of metal artifacts on CBCT images [15]. Although its image resolution is high, it may have an impact on visual judgment due to the visual fatigue of doctors or the effect of noise on the image. Besides, the early clinical symptoms of a cracked tooth are not obvious and easy to misdiagnosis. If the superficial fracture at initial diagnosis would be rapidly and effectively detected, it will undoubtedly be beneficial for clinicians to diagnose and develop subsequent medical treatment plans at the early stage of crack tooth symptoms. Therefore, the methods based on artificial intelligence (AI) as an auxiliary treatment to better facilitate the diagnosis of a cracked tooth may be a meaningful and helpful solution.

In recent years, with the development of AI and image processing technology, the image-based method implemented with deep learning was widely applied in crack detection in industry nondestructive testing for automation [16–18]. Among these methods based on deep learning, the image classification method is considered as one of the essential methods. The image classification-based methods essentially treat the crack detection problem as a binary classification problem (with or without cracks). Zhang et al. [16] proposed an automatic road crack detection method using ConvNet to classify 99 × 99 × 3 road image patches acquired by a low-cost smartphone, which shows outstanding performance compared with existing hand-craft methods. Cha et al. [17] proposed a 256 × 256 × 3 CNN classifier in combination with the sliding window algorithm, which improved the accuracy of crack detection to a level up to 98%. The work from Dorafshan et al. [18] had shown that CNN-based classification methods were superior in both detection speed and accuracy compared with the traditional common edge detectors (i.e., Roberts, Prewitt, Sobel, Laplacian of Gaussian, Butterworth, and Gaussian). Inspired by these achievements in applying CNN to crack detection in engineering, a ResNet50-based algorithm for the detection of cracked teeth is present in this article. To the authors' best knowledge, we introduce AI for the first time in the image detection of a cracked tooth and explore its feasibility for optical image detection of the cracked tooth. The proposed method here is combined with oral microscopic imaging of the tooth surface to suggest a rapid diagnosis and suggestion.

The following sections of this article are described as follows. Section 2 presents the proposed method and introduces the modified ResNet50 architecture and its detailed methodologies. Section 3 analyzes the training details of the CNN. Section 4 demonstrates the testing results of the trained CNN under various situations, and Section 5 is the conclusion of this article.

## 2. Methods

### 2.1. Overview of the Proposed Method

As reported in References [19] and [20], the ResNet50 model can be used as a useful and powerful tool for many biomedical applications, such as the detection of COVID-19 from chest X-ray images and the diagnosis in 12-lead electrocardiogram. In this article, a fine-tuning ResNet50 model was performed and tested for the automatic detection of superficial cracks in the cracked tooth.  Figure 1 shows a flow chart of using a CNN to detect cracks, which includes three steps: building a database of the cracked tooth, training the CNN model, and testing the trained CNN model. To train a CNN, a large number of raw images are taken from the surface of the cracked tooth, and these collected raw images are cropped into smaller images.

And then, the cropped images were manually divided into cracked and uncracked to generate a database containing 20,000 images. After that, the training set and validation set at a ratio of 4 : 1 are randomly selected from the database. Finally, these images are imported into a CNN for training and validation. The training process generates a CNN classifier, which can distinguish between images with and without cracks. Then, the trained CNN classifier (256 × 256 pixels) as a sliding window is used to traverse the entire original image (1920 × 1080 pixels) to identify the areas with or without cracks. In conclusion, by combining the trained CNN classifier and a sliding window algorithm, cracks in the tooth surface can be effectively detected.

### 2.2. Methodology

This section introduces the CNN architecture and its relevant theories for each layer of CNN in detail. A typical CNN usually consists of input, convolution, activation, pooling, full connection, and output layers. Besides, some other auxiliary operations, such as batch normalization and dropout, are often embedded in layers, which can speed up network training and reduce overfitting.

#### 2.2.1. CNN Architecture

Residual Network was a remarkable CNN proposed by He et al. [21] in 2015, which won first place in the ImageNet competition for the classification task. It was worth mentioning that the accuracy of the Residual Network even surpassed that of the human eye. Our work builds a CNN model by modifying the ResNet50 [21]. These modifications are as follows. First, the size of the input layer is modified from 224 × 224 × 3 to 256 × 256 × 3 to obtain more information when extracting features and can obtain faster efficiency in the subsequent sliding window process. Second, a fully connected layer with 2 units is added following the original fully connected layer and before the Softmax layer to achieve binary classification (with or without cracks). Finally, the dropout layer is used between the two fully connected layers to avoid the phenomenon of overfitting.

The architecture of ResNet50 in this paper consists of one 7 × 7 × 64 convolution layer, 16 residual blocks, and two full connection layers. Each residual block starts from a 1 × 1 convolution layer for dimensionality reduction, then a 3 × 3 convolution layer for feature extraction, and ends with another 1 × 1 convolution layer for increasing dimension to the same number of the input convolution layer in each block. And the identity shortcuts made the CNN more efficient, which solves the degradation problem due to the increase of the depth of a neural network. Besides, operations of batch normalization (BN) and rectified linear unit (ReLU) are also implemented after each convolution. The modified CNN architecture is shown in Figure 2.

#### 2.2.2. Convolution Layer

Convolution is an effective operation for extracting image features in deep learning. A specific number of 3 × 3 convolution kernels slide across the input tensor with an appointed stride. The weights of the convolution kernel and the values at the corresponding positions in the tensor are multiplied element by element. Finally, all the multiplied values are summed up, and bias is added to the summed values. And the weights in convolution kernels are updated in training using adaptive moment estimation (Adam). Usually, the all-zero padding method is adopted in the convolution operation to keep the input size consistent with the output size.  Figure 3 shows a convolution process with a bias of 0.

#### 2.2.3. Pooling Layer

Pooling is another core approach in CNN, and it is a kind of downsampling operation in the encoding path. The main purpose of the pooling layer is to decrease the data size after the convolution process, which can reduce the computational burden of the network and the risk of overfitting.

There are two types of pooling operations in general: max pooling and average pooling. Max pooling only selects the maximum value of the elements in the receptive field, whereas average pooling calculates the mean values. And Scherer et al. [22] have demonstrated that max pooling performed better than average pooling in convolutional architectures. Therefore, in this article, max pooing is adopted in all the pooling layers, as shown in Figure 4.

#### 2.2.4. Activation Layer

The activation function is a function with nonlinear, monotonic, and differentiable properties, which can give nonlinearity in neural networks. The activation functions can be divided into two categories, one is the saturated activation functions represented by sigmoid and tanh functions, and the other is unsaturated activation functions such as ReLU (Rectified Linear Units). ReLU solved the problem of gradient disappearance, which exists in saturated activation functions. Besides, it has a faster convergence rate because of the simpler derivation process [23]. ReLU is chosen in our model.

#### 2.2.5. Full Connection Layer and Softmax Layer

The full connection layer fully connects each neuron in the current layer with all neurons in the previous layer, and it usually connects the output of the last convolution layer or pooling layer, where the high-dimensional feature map extracted by the convolution and pooling operations expands into a one-dimensional vector. The function of the Softmax layer is to estimate a possibility for every class, which is connected after the full connection layer and located at the last layer of the CNN architecture.

#### 2.2.6. Subsidiary Layers

Overfitting has always been a common phenomenon in deep learning [17], and it easily occurs when training a network with a large number of neurons. Dropout operation is proposed to address this issue [24]. The function of dropout operation is to randomly delete some neurons in the hidden layers with a specified dropout rate. As a result, the trained network will be more generalizable due to the deceased dependence on certain local features. In our model, the dropout rate is set to 0.5.

BN is proposed by Ioffe and Szegedy [25] to accelerate training speed and improve model adaptability. The BN layer normalizes the current batch of data before the activation function to reduce the variability between samples, which prevents the data from being shifted and enlarged, thus effectively avoiding gradient disappearance and speeding up the convergence of the network.

## 3. Results

### 3.1. Building Dataset

The ideal dataset is prepared by the fresh extracted cracked tooth; however, it is really difficult to obtain intact. To build the dataset, it is necessary to prepare some simulated cracked teeth. Two hundred eighty-six fresh isolated human molars were collected from the Hospital of Stomatology, Sun Yat-sen University, and the Hospital of Guangdong University of Technology.

#### 3.1.1. Preparation of Cracked Tooth

First, soft scales and stains on the tooth surface were wiped with cotton swabs and rinsed with saline. Then used the microscope to pick out the isolated teeth with relatively intact crowns. Finally, 246 qualified isolated human molars were preserved in 10% paraformaldehyde.

In this study, the simulated cracked tooth was created based on the phenomena of thermal expansion and contraction. These samples were immersed in a tank of liquid nitrogen (−196°) for 24 hours. Then, the frozen teeth were immediately placed in boiling water for 5–10 minutes. The large temperature difference generated thermal stress, which further resulted in the microcracks in the sample. More details can be found in Reference [26].

#### 3.1.2. Image Acquisition

A total number of 800 images (1920 × 1080 pixels) were obtained by optical microscope with an industrial camera. The industrial camera parameters are shown in Table 1. First, 700 of these 800 raw images were randomly selected for training and validation of the CNN classifier model, and the remaining 100 raw images were used for the subsequent sliding window test. Then, these 700 raw images were cropped to a smaller size at 256 × 256 pixels and randomly divided into training and validation sets, at a ratio of 4 : 1. To obtain a CNN classifier with excellent robustness, these cropped images are captured under various situations and background features, as shown in Figure 5. On the other hand, the purpose of cropping images into images with a resolution of 256 × 256 is to meet the same size as the CNN input layer.

#### 3.1.3. Data Augmentation

The number of images in the dataset is 4,000 (the proportion of images with and without cracks is 1 :  1), which may cause the overfitting phenomenon in the classification task due to the limited dataset. Therefore, data augmentation is implemented in this study, which includes flip and contrast shift operations. After data augmentation, the total number of data sets is 20,000.

#### 3.1.4. Data Description

In the dataset prepared in this article, a total of 800 raw images of 1920 × 1080 pixels were taken from 286 fresh human molars using an optical microscope with an industrial camera. Among them, 700 randomly selected raw images were used for training and validation of the CNN classifier model, and the remaining 100 images were used for subsequent testing. The 700 original images used for training and validation were cropped to a total of 4,000 images with a smaller size of 256 × 256 pixels, and then expanded to 20,000 images through data augmentation (flip and contrast shift operations).

### 3.2. Optimizer and Loss Function

The loss function is one of the most significant mathematical components of a CNN model, which is defined as the objective function to optimize the model. Common loss functions include cross-entropy loss function, focal loss function, SoftMax loss function, and so on. To calculate the deviation between the predicted and actual values, cross-entropy is chosen as the loss function in this article, which is defined in equation (1):

(1) $$\begin{array}{c} L_{\text{ce}}=-\left[y\log\hat{y}+\left(1-y\right)\log\left(1-\hat{y}\right)\right], \end{array}$$

where *y* ∈ {0, 1} is the actual class probability and *y* ∈ [0, 1] is the predicted class probability.

To minimize the total loss during backpropagation, this article selected the Adam optimizer to update the model parameters. Among the numerous remarkable optimization methods like stochastic gradient descent (SGD), momentum method, root mean square prop (RMSprop), and so on. The Adam optimizer is considered as the most efficient and fastest method to narrow the deviations. It combines the advantages of the Adaptive Subgradient (AdaGrad) algorithm and RMSProp algorithm, which promote the gradients to converge at a commendable speed.

### 3.3. Training and Validating Results

The training process was accomplished on matlab2021b in a Windows system using a workstation configured with a high-performance GPU (NVIDIA Quadro p2200) and a CPU (Intel(R) Core (TM) i5-10500 CPU@3.10 GHz, RAM: 56 GB). The network is trained with a batch size of 32, a momentum of 0.9, and a weight delay of 0.0001 for 20 epochs.

The learning rate has a certain effect on the network's convergence speed and performance during training a CNN. To select a proper learning rate, the learning rates used in this article are set to 10^−1^, 10^−2^, 10^−3^, 10^−4^, 10^−5^, 10^−6^, and 10^−7^, respectively. Then, the network was trained for 10,000 iterations under different base learning rates and validated every 20 iterations. Recorded validation accuracies are shown in Figure 6. It can be seen that the validation accuracies and convergence speeds increase fast with the learning rate of 10^−3^, 10^−4^, 10^−5^, 10^−6^, and the final validation accuracy of them is all above 97%. The validation value of the cyan solid line with a learning rate of 10^−4^ seems to be the best learning rate, because the value of the accuracy increased fastest. However, the upward trend of the training process is relatively unstable, and the ultimate accuracy converged to 99.03%, which is lower than the learning rate of 10^−5^ (99.12%). In the largest learning rate of 10^−1^, the accuracy maintains at about 50% from start to end, which indicates the training of the CNN is nonconvergent. When the learning rate decreases to 10^−2^, the convergence speed becomes low and achieves the ultimate validation accuracy of about only 88.25%. It can be seen that the minimum learning rate 10^−7^ performed worse, which may be caused by overfitting. The key finding from the training results demonstrates that a proper learning rate can make a CNN converge faster and obtain higher validation accuracy during training. As a result, the learning rate 10^−5^ is selected as our model hyperparameters.

Figure 7shows the feature images of the first and the tenth convolution layers, and 64 feature images were obtained for each layer. As shown in Figure 7(b), some feature images show the blurred outline of the crack. As the convolution operation continues, some extra interference is filtered out. The ideal feature of the crack is extracted from some feature images in Figure 7(c).

## 4. Discussion

To test the performance of the trained and validated CNN from the previous section, 100 raw images with 1920 × 1080-pixel resolutions that are not selected for training and validation processes are used in the testing. Notably, the trained and validated CNN framework shows nearly the same performance without any degradation of the accuracy, even though different images (normal, the presence of other dental diseases, stained tooth surface) are used for testing.

In the sliding testing results, the regions in original images with cracks are defined as positive regions, and the opposite are negative regions. Meanwhile, if the trained CNN detected and classified the positive and negative regions correctly, then these areas are defined as true-positive and true-negative regions, otherwise false-positive and false-negative regions, respectively. It is worth mentioning that one of the authors in this article is a professional dentist, who have checked the data annotations of cracked tooth. The testing accuracy of each image is calculated using equation (2):

(2) $$\begin{array}{c} \text{ Accuracy}=\frac{\text{TP}+\text{TN}}{\text{TP}+\text{TN}+\text{FP}+\text{FN}}. \end{array}$$

Among them, TP, TN, FP, and FN represent the number of true-positive, true-negative, false-positive, and false-negative regions in the tested images, respectively.

Figure 8 depicts the testing accuracy of 100 raw images. Inspiringly, the average accuracy of them is 90.39%, which is close to the validation accuracy. Besides, the performance of the trained CNN is still remarkable even though different images under various conditions are used for testing, and it takes about 10 seconds to test each image.

This article selects and presents some representative tested images under various conditions, where the false-positive and false-negative regions are highlighted as green and red colored square illumination boxes, respectively, as shown in Figures 9–11.  Figure 9 shows images of normal tooth surfaces with different degrees of the crack size of microcracks. The testing results are generally encouraging where most cracks are detected correctly. Especially in Figure 9(b), the trained CNN can successfully detect the image with extremely thin cracks that are difficult to be observed with visual inspection. However, image distortion may affect the accuracy. In the image that has normal cracks and fine cracks in Figure 9(c), three false-negative regions are distributed at the periphery of the raw image center due to the image distortion in the thin crack region. It may be because distorted images result in poorly characterized cracks, which prevent them from being recognized by the network. Crossed cracks may reduce detection accuracy to some extent. For example, in Figure 9(e), all cracks in original images are still detected correctly, although there is one false-negative region in the images from blurred and distorted surfaces. On the other hand, the misjudgments of forming false-negative regions are these cracks at the edge of each sliding window, because the image would be continuously smaller when the input image passes through CNN, resulting in less chance for the cracks at the edge of the image to be recognized by the network than the cracks in the middle of the image.

To learn the effect of CNN on illumination, two images with light spots of different degrees of crack size were tested. It turns out that strong light may cause errors in crack detection, as shown in Figure 9(a) and 9(d). In Figure 9(a), normal cracks in original images are all detected correctly. In Figure 9(d), there are two false-negative regions with extremely tiny cracks in the images from strongly lighted tooth surfaces. And further addition of images about the corresponding samples of overexposed images to the dataset may tackle the above problem.

To explore the sensitivity of the network to the disturbances of other diseased tooth surfaces (cavities, dental plaque, etc.). In Figure 10(a), in the image of tooth surface with cavities, only one false-negative region with a thin crack exists. In the image of the surface with dental plaque in Figure 10(b), there are two false-negative regions from the uneven surface. The results showed a good generalization of the proposed CNN.

To examine the robustness of the trained CNN further, three images with stained tooth surfaces are chosen in Figure 11. It can be clearly seen from the testing results that most of the stains do not affect the judgment of the proposed CNN, but those stains with a shape of near-strip would be labeled as false-positive regions by the CNN. Under the condition of normal cracks in the stained tooth surface image in Figure 11(a), only one false-positive region exists. This type of image includes complex cracks as shown in Figure 11(a) and 11(b) and false-negative region with blurred areas with cracks are not detected by the CNN. In the image with crossed normal and thin cracks in Figure 11(c), the testing results provide a desirable testing accuracy of 89.29% with only one false-negative region and two false-positive regions.

In a nutshell, the proposed method presents robust performance and strong adaptability in tooth crack detection under various conditions of the raw images, which will provide satisfactory effectiveness in the real world. Using binary classification CNN to realize the automatic detection of cracks in the cracked tooth may definitely provide worthy or amazing diagnostic methods with more intelligent, automated, and specialized solutions.

## 5. Conclusion

This article used CNNs with a sliding window algorithm to detect cracks from optical images. The CNN architecture of binary-class output for crack detection was designed by modifying the classic ResNet50. Eight hundred images with 1920 × 1080-pixel resolutions acquired by an optical microscope with an industrial camera were used to train, validate, and test the CNN where all of the images were taken from the simulated cracked tooth. To build the training set and validation set, 800 images were cropped into 20,000 smaller images of 256 × 256-pixel resolutions. To choose the best learning rate according to validation accuracy, seven different learning rates were set during training the CNN. By comparing the training results under different base learning rates, the learning rate of 10^−5^ was chosen with the highest validation accuracy of 99.12%. Combined with a sliding window algorithm, the trained CNN was tested on 100 raw images under various situations, such as the stained, overexplosion, affected by other diseases, etc. Encouragingly, the average testing accuracy reached 90.39%.

The purpose of the presented classification-based CNN combined with a sliding window algorithm is to propose an image processing method to assist clinicians in the diagnosis of cracked tooth, aiming at helping them to make diagnostic decisions and proposing relevant suggestions and recommendations. The current method was initially explored and verified for the detection of cracks on the tooth surface, and it can be widely extended to other imaging tools (e.g., CBCT, Oral X-rays, etc.) in the following study. For example, the proposed method can also be used for the detection of root fracture if associated with CBCT imaging.

Even though we have achieved encouraging results by testing the simulated cracked tooth under various conditions, there are still some limitations of the proposed method. First, the construction of the dataset in this article is based on the simulated cracked tooth, which may affect the accuracy of the clinical detection of cracked tooth. Second, the real oral cavity is more complex, factors such as lighting can have an impact on the quality of the image, which may increase the difficulty of taking clear optical photographs for subsequent image analysis. Third, the method currently detects some superficial cracks on the teeth. More research can be done in combination with CBCT and oral X-rays to detect other types of cracked tooth, for example, VRF (a fracture that originates from the coronal (enamel) or apical (root) portion of the tooth and usually extends faciolingually). In a nutshell, this article created a dataset of cracked teeth and conducted a subsequent AI-based method to detect the cracks on the teeth. In the next step, according to the oral environment and different imaging schemes, some improvement studies will be conducted on hardware design and software optimization for multiple aspects of the network, including the real-time ability, accuracy, and clinical applicability.

## Figures and Tables

**Figure 1:** Flow chart for detecting cracks the proposed method. The trained CNN classifier (256 × 256 pixels) can effectively identify the areas with or without cracks in raw images (1920 × 1080 pixels) by combining the sliding window algorithm.

**Figure 2:** The architecture of the proposed CNN which is modified based on the classic ResNet50. Two major changes are as followed. First, the size of the input layer is modified from 224 × 224 × 3 to 256 × 256 × 3. Second, a fully connected layer with 2 units is added before the Softmax layer.

**Figure 3:** Illustration of the convolution process with bias of zero.

**Figure 4:** The illustration of the max pooling process.

**Figure 5:** Sample display of partial dataset. Some cracks in images under various conditions (stained, overexplosion, affected by other diseases).

**Figure 6:** Validation accuracies under seven different learning rates. Lr represents the base learning rate.

**Figure 7:** Visualization of features: (a) raw images; (b) feature visualization after the first convolution (64 images); and (c) feature visualization after the 31st convolution layer (64 images).

**Figure 8:** Testing accuracies of 100 new images, and the average accuracy is 90.39%.

**Figure 9:** Testing results for image containing different types of cracks: (a) normal cracks; (b) tiny cracks; (c) normal cracks and thin cracks; (d) tiny cracks and lighting spot; and (e) crossing cracks. The red arrows point to the crack.

**Figure 10:** Testing results for image containing other diseased tooth surfaces. (a) Cavities exist on the tooth surface with tiny cracks; and (b) tooth surface with dental plaque with normal cracks. The red arrows point to the crack.

**Figure 11:** Testing results for image containing stained tooth surfaces of different types of cracks: (a) normal cracks; (b) normal crossed cracks; and (c) normal cracks and tiny cracks. The red arrows point to the crack.

**Table 1:** The industrial camera parameters.

Product model	Specification	
USB3.0 industrial camera	Effective pixels	16 million
	Resolution	1920 × 1080@30FPS
	Sensor	MN34120
	External dimension	47 × 35.8 mm
	Size of pixel	1.335 × 1.335 μm

## Data Availability

The datasets generated during and/or analyzed during the current study are available from the corresponding author on reasonable request.

## Abbreviations

PR: Periapical radiography
CBCT: Cone-beam computed tomography
CNN: Convolutional neural network
AI: Artificial intelligence
CT: Computer tomography
Micro-CT: Micro–computed tomography
OCT: Optical coherence tomography
MRI: Magnetic resonance imaging
VRF: Vertical root fractures
AAE: The American Association of Endodontists
BN: Batch normalization
ReLU: Rectified linear unit
Adam: Adaptive moment estimation
SGD: Stochastic gradient descent
RMSprop: Root mean square prop
AdaGrad: Adaptive subgradient.
